# The Impact of Online Learning System on Students Affected with Stroke Disease

**DOI:** 10.1155/2022/4847066

**Published:** 2022-02-07

**Authors:** Sobia Wassan, Chen Xi, Tian Shen, Kamal Gulati, Kinza Ibraheem, Rana M. Amir Latif Rajpoot

**Affiliations:** ^1^Business School, Nanjing University, China; ^2^School of International Education, Nanjing University of CM, China; ^3^Amity University, Noida, Uttar, Pradesh, India; ^4^Stratford University, Virginia, USA; ^5^Department of Computer Science COMSATS University Islamabad, Sahiwal Campus, Pakistan

## Abstract

Stroke, also known as a cerebrovascular accident, is a medical emergency that causes temporary or permanent behavioral dysfunction in people. Sleep deprivation affects our brains in a variety of ways. The advantages of sleep much justify the risks of not having enough sleep. Sleep deprivation (SD) includes a variety of factors, including prolonged awake. Neuroimaging investigates SD's impact on attention, working memory, mood, and hippocampal learning. We analyzed how this data enriches our mechanistic understanding of these alterations and the clinical illnesses linked with sleep disruption. We have used Cronbach's alpha to test the reliability of a scale, so we then have 19 individual attributes responding to 174 participants via survey. The evaluated result shows the reliability statistics; the value for Cronbach's alpha is .962, which is very excellent as it reaches 1. So, there is very strong reliability. If the value falls under .6, we look back to the mean and standard deviation table and remove the attribute with low values for mean or standard deviation and try the remaining attributes. Cronbach's alpha tells us which attribute or item to delete to increase the reliability, and we also have analyzed the correlation among the class students while watching the same video lecture. We have collected data for at least ten students watching the same video using a webcam. Once the data is collected, we then have applied some correlation techniques to determine the class students' behavior towards the same video lecture. This way, we can see the overall behavior of the class upon a specific video lecture. The study further reveals that subjective happiness is influenced by its efficiency, entertainment value, and effectiveness. Does the research offer an original emphasis on analyzing how does lack of sleep affect our brains? Sleep loss frameworks are minimal compared to the benefits of sleep.

## 1. Introduction

Our cognitive and emotional capacities are negatively affected when we do not get enough sleep. What alterations in the brain are causing these abnormalities? In this article, the authors [1] explained what do these changes reveal about the widespread relationship between sleep disturbance and a variety of neurological and mental disorders? [1]. The authors [2] explained that there are at least three reasons to accurately describe how SD impacts the human brain. One must first determine whether brain networks are prone or resistant to the special effects of sleep deprivation and how SD-induced changes in activities or functional connections justify the deleterious changes in behavior related with SD. Sleep deprivation does not only refer to sleeplessness and the associated behavior's, though. Rather, sleep deprivation is a combination of several harmful causes, including prolonged alertness and lack of sleep. It is thus inadequate to learn about the functional advantages of sleeping and then learn about the neurological and behavioral alterations that occur when sleep is lacking. Second, all significant neurological, including schizophrenia, Alzheimer's disease, and other serious neuropsychiatric disorders, and anxiety disorders have concomitant sleep disturbance. Attention, which is required for continuous goal-directed behavior, is one cognitive capacity that is particularly vulnerable to sleep deprivation. Due to increased sleep pressure, attentional activities decline in a dose-dependent way as the sum of time spent wakeful grows [3]. In this article, the authors state that “lapses” or “microsleep” is a prototypic deficit on such tasks that entail reaction failure that reflect errors and omissions [4]. The authors explained that increased sleep propensity and instability of waking neurobehavioral processes are connected to poor cognitive performance and severe social, economic, and health-related implications. Sleep deprivation has been shown to impair a variety of cognitive processes, including attention, memory, and learning [5]. In this article, the aim of this analysis is on sleep loss; it is worth noting that daily clock alertness signals interact with SD to cause attentional impairment that increases exponentially with increasing awake time [6, 7]. The behavioral repercussions of these brain alterations include difficulties focusing on a single input while disregarding distractions [8, 9]. It is less clear why some people are more or less susceptible to these attentional problems after SD than others. A clearer understanding of how severe SD affects brain function linked to attentional activities is developing. When performing attentional tasks, SD reduces fMRI signals in the DLPFC and temporoparietal sulcus [10]. Reduced activity in the DLPFC and temporal and parietal sulcus has a role in attentional performance failure once again [11]. Nonetheless, the authors state that the total time spent awake predicted attention deficits in both acute and chronic partial sleep deprivations [2].

### 1.1. Awakening with Sleep Deprivation

SD enhances amygdala activity (red) and decreases amygdala–MPFC connectivity (blue). SD alters the salience-detection network's sensitivity to emotional signals ranging from adversely (red) to neutrally (blue) to positively (green) (red). The capacity to discriminate between emotion (red vertical line) and neutral (blue vertical line) stimuli is enhanced during sleep (left graph). Reducing one's capacity to discern between emotion salience levels may be reduced by using SD (right graph) (short vertical difference line). The salience-detection network misidentifies a seemingly neutral input (blue line) as emotional, leading to skewed emotional judgments of neutral stimuli. These central brain alterations, together with impaired peripheral cardiac nervous system input of visceral bodily information, may result in erroneous or missing emotional expression. Experiments reveal that people who are sleep deprived cannot recognize emotive faces on a computer and so cannot correctly duplicate their emotional expressions. Part A is from REF with permission [12] (Elsevier).

Under SD circumstances, adequate persistence of DMN activity is seen throughout working-memory task execution [13]. On the other hand, the amount of abnormal, on-task DMN activity predicted the intensity of sleep-deprived people's working memory deficits [14] (Figure 1). A common process causing SD-induced attentiveness and memory issues might be insufficiently gated on-task vs. off-task network control. Because the thalamus is involved in cortical arousal, changes in thalamic activity and connectivity can calculate memory losses under stressful conditions (SDS). An improved link between the thalamic DMN and the hippocampus is associated with increased subjective exhaustion in sleep deprivation, as well as a worse performance in working memory tasks [15].

A literature review appears in Section 2, a methodology appears in Section 3, the results and discussion appear in Section 4, and the conclusion and future research appear in Section 5.

## 2. Literature Review

Cognitive changes are quite prevalent (80%). The most prevalent issues are as follows: memory focus processor speed changes in selective attention and visual-spatial/perceptual processing are common. It might be evident (aphasia, neglect) or subtle (e.g. intellectual underfunctioning and visuoperceptual difficulties). In contrast, a higher thalamus-precuneus connection predicts better working-memory recovery in SD than in sleep-rested. This data supports the concept that in SD, partially recovering specific behaviors is possible due to compensation neural activity in the brain [16]. The authors explained that during concentration activities, thalamic activity fluctuates [17]. The combined impact of nap times and nocturnal sleep on stroke risk is unknown. The authors' study used data from the large cross-sectional and cohort investigation to corroborate this association [18]. Sleep efficiency declines with age, affecting the quality of life. Also, a stroke that occurs while sleeping might be fatal to an aged person. So, real-time health monitoring is critical for stroke detection. Material(s)/Method: Smart IoT sensors integrated into mattresses, wearable gadgets, and clothing record and physiological factors such as brainwaves, sleep movement, and muscle activation. Sleep monitoring devices assess sleep quality and detect sleep disorders [19]. To address the influence of continuous sleep on cerebral apoplexy in Chinese people, the authors' research demonstrates that persons with durative somnipathy have more adverse occurrences [20]. Poststroke tiredness is a typical consequence of stroke that affects the quality of life. Although numerous therapy techniques have been investigated in the past decade, the risks for PSF remain unclear. This meta-analysis sought to identify PSF risk factors, particularly clinical and social associated with an increased risk, that may be prevented [21]. After a stroke, up to two-thirds of individuals develop OSA. These individuals had poorer short-term sickness, cognitive and functional recovery, and long-term death rates than those without OSA. Detecting OSA and controlling it with positive airway pressure (PAP) are key therapeutic aims after a stroke [22]. People who have had a stroke often have trouble sleeping. Poor sleep is linked to a worse quality of life, and more research is required on the long-term effects of stroke on sleep. This study compared the sleep habits of chronic stroke patients with those of nonsurvivors. The authors looked at mood and activity as possible sleep correlations [23]. At the beginning of the study, 95,023 Chinese volunteers who had never had a stroke were surveyed (2006-2007). The authors explained that based on sleep duration, the Cox proportional models were used to calculate stroke hazard ratios and confidence intervals [24]. Stroke rehabilitation patients in Canada were monitored for two weeks to determine their activity levels and sedentary time [25]. The results of a study published in the *Journal of Sleep Research* suggest that chronic sleep deprivation can lead to cumulative waking neurobehavioral impairments [3]. An attack on the brain known as a stroke occurs when the “unexpectedly disruption of blood supply.” The blood flow to a portion of the brain may have been unexpectedly halted or a cardiovascular system ruptured. The term “wake-up stroke” refers to a condition in which a patient wakes up with symptoms that have never been seen before they went to sleep [26]. The results of their study were published in the *Journal Sleep Research*, where they describe how awake neurobehavioral and physiological processes are measured and compared to those of people who do not sleep at all [2]. The purpose of this research is to examine if poststroke urine incontinence (UI) affects one-year outcomes in terms of attention and cognitive processing speed [27]. Physical therapists who treat persons with chronic stroke in the community were the focus of the research. Professionals caring for long-term stroke survivors may benefit from the findings of this research in [28]. In this article, the authors stated that three teaching hospitals in the United Kingdom conducted a study comparing aged care, general medical care, and stroke care [29]. Deglutition seems to be more significant than swallowing postischemic impairment. A prompt swallowing rehabilitation may enhance and speed up the recovery of patients with apparent clinical, psychological, and economic benefits. An Italian rehabilitation center has already been treating a patient with ischemic illness and stroke at Udine Civil Hospital since 1989 [30]. Tissue plasminogen activator (TPA) injections and thrombectomy were previously restricted to 4.5 and 6 hours, respectively [31]. What happens to our brains when we do not get enough sleep? Frameworks for assessing sleep loss are few in comparison to the positive effects of sleep. Sleep deprivation (SD) is not only about the lack of sleep and the associated advantages; rather, it is also about a variety of other things, including prolonged awake. Neuroimaging studies are used to examine the special effects of SD on attention and working memory, positively and negatively reaction, and hippocampal learning. There are recognized changes in cognition and emotion related to sleep disturbance, This data can help us develop a mechanistic understanding of these changes, in addition to understanding how sleep disruptions cause clinical disorders. We have used the Cronbach's alpha to test the reliability of a scale, so we have 19 individual attributes that have been responded by 174 participants via survey. The evaluated result shows the reliability statistics; the value for Cronbach's alpha is .962, which is very excellent as it reaches 1.

## 3. Methodology

A stroke often causes cognitive and memory damage. A year after a stroke, 30% of people acquire dementia. Stroke impairs attention, cognition, language, and direction. The suggested research approach includes phases of data collection and analysis. Comparison of existing work and a comparison of why we have selected this topic will also be elaborated in detail. The research methodology for visual attention is presented in Figure 2. These data were collected through the use of multimedia software and instruments within the e-learning environment. During the data collecting time, we focus on student attention scores by capturing the face, the eyes opened and the eyes closed in the form of photographs to assess students' interest. After collecting data in the form of photographs, we analyze students' comprehensibility using the developed app. To assess the results' validity and correctness, a comparison is made between the software and manual observation of students in the e-learning environment. The methodology steps are as follows:

- Firstly, the data is collected as a CSV file whenever the student watches the lecture using the C# application's webcam, and it is logged in the system
- The study of datasets based on attentiveness scores shall be retained
- The correlation will be made among all the students of the class with some graphical representation

Whenever we want to assess the students' attention, we collect the student data from the webcam in the first step. The information is gathered while the student watched the lecture. We are going to give an example of the method for collecting data. Let us imagine S1 is a student viewing a video lecture, and we want to gauge S1's attention using facial expressions. S1 viewed the video lecture for this purpose; meanwhile, his/her computer's webcam is on. Our C# application runs behind the scene and collects each image where the student's face is in front of the webcam. When a webcam sensor detects a face or a C# application sensor detects a student's facial features, the C# app saves the photo to the computer system.

Later, we develop the results and experimentations, the C# application converts a large picture to a small 64 × 64-dimensional image, transformed into a 96 dpi 8-bit grayscale image. Switching the image to grayscale, after that on, helps to identify facial expressions more easily and quickly.

The C# program also enhances the image quality before saving it to a computer system. The front is, however, detected by the Haar Cascade Classifier accessible in C#. We can see in the image below how the images look when they are stored on the system.  Figure 3 shows sample photos of 10 students watching the lecture.

We are implementing the detection and saving of the face. Meanwhile, we are preparing a column that has been saved to a CSV file that the C# framework can generate automatically. ScoringDataNumber.csv is the name of the file, and the number reflects the user ID who is watching the same video lecture. Figures 4 and 5 display a preview of the dataset file.

### 3.1. Number of Faces

This section specifies the number of faces in the webcam image. For detecting the number of faces within a picture, the C# app uses the Haar Cascade Classification.

## 4. Actual Eyes

For example, when two sides are detected in the actual picture frame, the values in this column are 4. But if only one face is identified in the current image frame, the value is two. The attentiveness of the current face will later be determined exactly.

### 4.1. Detected Eyes

This column reflects the current image's eyes; its value maybe 0, 1, or 2.

### 4.2. Opened Eyes

For example, if one eye is opened on the detected face, the value is 1; if both eyes are opened, then the value is 2.

### 4.3. Closed Eyes

This column tracks the closed column's reverse values, because if one eye is closed in the current face recognition, the value is 1 and, when both eyes are closed, the value is 0, etc.

### 4.4. Eye Detection Error

This column records the eye-tracking error; for example, if multiple faces were observed in the existing frame and the numbers of eyes identified were one or null, the eye identification error would be 1 and 2, so if one eye were spotted, the number of eyes detected would be 2. The detection error method is seen below.

(1) $$\begin{array}{c} \text{Eye detection error}=\text{actual eyes}–\text{detected eyes}. \end{array}$$

### 4.5. PFPS

This column shows the number of frames per second processed.

### 4.6. Attentiveness

This column records the score of attention using the formula given:

if (numberOfFaces != 0)

attentiveness = ((0.5 ∗ numberOfFaces ∗ 2 / actual Eyes) + (opened Eyes / actual Eyes ∗ 0.5));

else

attentiveness =0;

While using the above formulas, the value remains o.5 or 0.75 or 1 for attention.

### 4.7. Attention Level

This attribute is very important as it tells us how sleepy a student is if the attention value is 0.5, 0.75, or 1, this value is considered satisfying. This value is considered an attention level in this column.

## 5. Validating the Student's Behavior towards Online Learning

Personalized learning is part of learning for hundreds of years. In the past, when the facilities in the education field were so less, the number of schools was too less; people learn their prior knowledge from home or any intellectual person from the family. After this, thousands of schools open, and students get their education by themselves. They go to school and get an education, but many students cannot afford the fees and expenses. For this, they go for a job and mostly prefer online learning or personalized learning. This type of education they can get when they are free from their jobs. In online learning, the student's attention level is how much he is attentive when he takes the lecture. Due to the coronavirus (COVID-19) worldwide, a pandemic situation spread in today's time. More or less, everything has been stopped worldwide; as per condition, all schools, colleges, and universities are helpless. They all are intended to give online education, as the big issue is that our students are not used to taking online classes because their reflexes and attentional level are not as high. So, in this research work, we measure the student's attention level; we will check the student's behavior. For this, we will generate a survey for the students of Pakistan. Because in Pakistan, the literacy rate is almost half of the population; also, they are not used to online leering and search for things from the Internet and research work.

### 5.1. Google Analytics Visualization

In this section, we have visualized the population's detail, which is involved in the survey. We have to take the survey from 174 genders from Pakistan. The ratio of male and female is as shown in Figure 6, where the 64.9% population from the male side and 35.1% are females.

In Figure 7, we have shown the educational level of the population involved in this survey. There are four major categories: higher secondary, undergraduate, postgraduate, and Ph.D.

Figure 8 shows the ratio of the prior information of the population relating to knowledge about the Internet. As in online learning, the knowledge related to the Internet is more important. So, we have seen that 39.7% have good knowledge and 5.2% have less knowledge about the Internet.

Figure 9 displays the average rate that how much time in a day you have spent on the Internet. So, we have analyzed half of the population spends more than four hours on the Internet in a day.

Figure 10 shows how many students are taking online classes in a day, week, and month. Our analysis showed that 56.9% have taken online classes daily.

In Figure 11, we have asked students which platform they have mostly used for online learning: our query regarding the most rated online learning platform like EdX, Coursera, NPTEL, or Udemy. We have evaluated that 86.2% population is not encouraging these all-top-rated platforms. They want to learn online from their institutes or the Internet [32].

Figure 12 shows that 50.6% of the population prefer to learn from the Internet, and they do not want to pay their institutes or coaching centers, because they want to learn free of cost [33].

Figure 13 shows the sample screenshot of the dataset which we used in our analysis; in the dataset, we have asked multiple question from the students. Therefore, in our analysis, we cannot use these questions as it is in SPSS tool. Thus, we have converted them in a short form variable that can easily generate the results. So the short form abbreviated questions are as follows: Internet Hours, OnlineClassesHelpLongRun, OnlineClassesWillImproveLearning, PersonalSuccessByOnlineClasses, OnlineClassesHelpBoostSkills, OnlineClassesAreSimpleToUse, OnlineClassesMoreFlexible, FavorableAttitudeTowardsOnlineClasses, OnlineClassesImpactsPositivityOnMe, OnlineClassesUseIsTrend, IntendToUseOnlineClasses, IncreaseOccurracneOfOnlineClasses, OnlineClassesWillEnhance, OnlineClassesConsistentWithDevices, SystemUseWillBoostMyLearning, OnlineClassesMatchesWithOldSystem, TryAnyFunction, IknowBefore, and TryTechnologyToEvaluate.

## 6. Results and Discussion

### 6.1. Overview

Our results from the extracted dataset that we discussed earlier were presented in this section; so there are three levels of attention:

- Sleepy
- Satisfactory
- Attentiveness

Image 14 showed the attentiveness and attention level results of the ten students. In this figure, we tested the 10 students' attentiveness and attention level, which is the display with the name S1 to S10.

### 6.2. Student1 Attentiveness and Attention Level

Student1 (S1) remains the most attentive when the sleepy attention level is the second-highest in the graph. And then, the student's attention level turns to be satisfactory for very little time compared to the attentive attention level.

### 6.3. Student2 Attentiveness and Attention Level

Student2 (S2) seems very attentive, as we can see in the picture; attentive attention is much higher than satisfactory and sleepy.

### 6.4. Student3 Attentiveness and Attention Level

Student3 (S3) is attentive, and then, its graph is a little bit satisfactory; then the student is sleepy. Therefore, we can say the student has almost 60% of attention to be attentive here.

### 6.5. Student4 Attentiveness and Attention Level

This student is sleepy, and very little proportion seems to be satisfactory. Therefore, we can say this student has very low interest in the lecture.

### 6.6. Student5 Attentiveness and Attention Level

Student5 (S5) is like student4 (S4); this student is also sleepy almost all the time, so the student seems the least interested in the lecture, or he/she is sleeping and not watching the lecture properly.

### 6.7. Student6 Attentiveness and Attention Level

Student6's (S6) behavior is almost the same as student5's because this student is almost sleepy and satisfactory for a very short interval.

### 6.8. Student7 Attentiveness and Attention Level

Student7's (S7) graph shows that he/she is a little bit satisfactory, and most of the time, the attentiveness level is sleepy, so we can say this person is sleepy as well and not interested or not watching the lecture properly.

### 6.9. Student8 Attentiveness and Attention Level

Student8 (S8) is a little bit satisfactory and, most of the time, sleepy, so this student is also not watching the lecture properly, or we may say that the student is not interested in the lecture.

### 6.10. Student9 Attentiveness and Attention Level

Student9 (S9) is a little bit interested in the lecture because some of the graphs show satisfactory and attentive behavior. Again, the student gets sleepy for almost half of the time than satisfactory and attentive attention.

### 6.11. Student10 Attentiveness and Attention Level

Student10 has mixed behavior like in [34]. As we can see, the graph has a considerable bar for being attentive and satisfactory now. Comparing both attention levels with the sleepy attention level is also very strong; this may conclude that student10 S10 and was about 0% interested in the lecture. Before we conclude overall behavior, we might consider that our eyes get closed after a specific time interval, so every graph has some kind of natural biases. However, by considering that face, we can even then see considerable sleepy behavior. We can conclude here that the lecture topic is boring, or the students are not interested in watching this specific lecture for some reason. Now it is up to the teacher; he/she should take some feedback from the students to improve the lecture or ask them to watch the lecture more attentively if there is no problem with the lecture content or video quality, as shown in Figure 14.

### 6.12. Correlations

The following table shows the correlations among the ten students. So, any significant value, which is less than 0.05, shows a strong relationship. The significance value of S1and S2 is 0.025, so S1 and S2 have a strong relationship, and we have also seen it above in the graph analytics.

If we compare the correlation between s4 and s2, then the significance value S4 is .705, which is very large than 0.05, so there is no good relation between s4 and s2, which is also seen well in the graph analytics above. Likewise, we can check all the pairs, and every pair will support the graph analytics results discussed above and shown in Tables 1–3.

### 6.13. Reliability Scale: All Variables by Cronbach's Alpha Using SPSS

Cronbach's alpha is a test of the reliability of a scale, we have 19 attributes so we have 19 individual attributes responding to participants via survey. Cronbach's alpha can be used to test the reliability of the scale when we have a series of items/attributes; in this case, we have 19 attributes. We can see only 4 rows are excluded or miss some values while there are 170 cases considered for the results, as shown in Table 4.

#### 6.13.1. The Procedure Is Deleted List-Wise Based on All Variables

Table 4 shows the mean and standard deviation of the attributes used for further interpretations. The following table is very important as it shows the reliability statistics; the value for Cronbach's alpha is .962, which is very excellent as it reaches 1. Thus, there is very strong reliability. If the value falls under 6, we look back to the mean and standard deviation table and remove the attribute with low values for mean or standard deviation and try the test for the remaining attributes, as shown in Tables 5–7.

The total item statistics 2^nd^ column tells us the value for Cronbach's alpha if a specific item or attribute is deleted. For example, if we delete the first attribute and apply Cronbach's alpha on the remaining items, the reliability scale value will be 7.16. In this way, we can highlight each attribute's significance. Hence, if an attribute does not affect the value of reliability, we can go ahead and delete that attribute. So, Cronbach's alpha tells us which attribute or item to delete to increase the reliability. Still, in our case, we have luckily chosen the attributes which are best already, so we will not delete any attribute, as shown in Tables 8 and Table 9.

## 7. Conclusion

Medical emergencies such as strokes, which are also known as cerebrovascular accidents, can induce behavioral dysfunction in people. Sleep deprivation affects our brains in several different ways. When compared to the advantages of sleep, sleep loss frameworks are minimal. Many factors contribute to sleep deprivation (SD), including being awake for an extended period. Neuroimaging studies the effects of SD on attention, working memory, mood, and hippocampus-based learning. To assess biosignaling/bioimaging data acquired from the patient, automated diagnostic techniques are generally favored. In this research, we explored the association between watching the same lecture and students' results. For ten students watching the same video, we collected data via a webcam. We also implemented graph analysis and correlation methodology after the data was collected to determine the class students' behavior towards the same video lecture. We noticed that most students were not interested in this video lecture. Still, the teacher can ask the students to view the lecture more carefully. If there is any problem with the lecture's quality or the topic is confusing or boring, the teacher can give the lecture to the students again and maybe take some necessary action. The alpha of Cronbach showed a strong correlation between the attributes/questions that we asked in our survey, and we will use this survey to prepare for online class evaluations.

## 8. Future Work Limitations

The purpose of usage may have been determined by certain considerations, such as prior experience required to take a specific course, not included in the analysis. There will also be further variables in prospective experiments, and the connections between them should be established or the indirect influence of the variables included in the current model tested. This work is limited to survey data in the future.

## Figures and Tables

**Figure 1:** Sleep rested vs. sleep-deprived.

**Figure 2:** Research technique for students' visual focus.

**Figure 3:** The sample pictures of 10 students while watching the lecture.

**Figure 4:** The sample screenshot of student1 for measuring the attentiveness while taking the online lecture.

**Figure 5:** The attentiveness level of the ten students while taking the online lecture.

**Figure 6:** The percentage of the population involved in the survey.

**Figure 7:** The percentage of the education level of the population involved in the survey.

**Figure 8:** The percentage of the knowledge rate population involved in the survey.

**Figure 9:** The percentage of how much time students spend on the Internet in a day.

**Figure 10:** The percentage of how often students take online classes.

**Figure 11:** The percentage of the ratio of the top-rated online platforms.

**Figure 12:** The percentage of how much fee students want to spend for online classes.

**Figure 13:** The sample screenshot of the dataset for student behavior related to the online classes.

**Figure 14:** Visualization of 10 students' attentiveness by attention level.

**Table 1:** Descriptive statistics.

	Mean	Std. deviation	*N*
S1	.8772	.21086	851
S2	.9239	.18474	851
S3	.8481	.21810	851
S4	.5247	.07845	851
S5	.5320	.08872	851
S6	.6366	.19230	851
S7	.5400	.09166	851
S8	.5138	.06207	851
S9	.5006	.01211	851
S10	.5000	.00000	851

**Table 2:** Correlations^d^ (a).

		S1	S2	S3	S4	S5	S6
S1	Pearson correlation	1	.077^∗^	.086^∗^	.032	-.045	.006
	Sig. (2-tailed)		.025	.012	.347	.189	.857
S2	Pearson correlation	.077^∗^	1	.058	.013	.041	.123^∗∗^
	Sig. (2-tailed)	.025		.092	.705	.230	.000
S3	Pearson correlation	.086^∗^	.058	1	.108^∗∗^	-.011	.010
	Sig. (2-tailed)	.012	.092		.002	.758	.779
S4	Pearson correlation	.032	.013	.108^∗∗^	1	.087^∗^	.044
	Sig. (2-tailed)	.347	.705	.002		.011	.196
S5	Pearson correlation	-.045	.041	-.011	.087^∗^	1	.118^∗∗^
	Sig. (2-tailed)	.189	.230	.758	.011		.001
S6	Pearson correlation	.006	.123^∗∗^	.010	.044	.118^∗∗^	1
	Sig. (2-tailed)	.857	.000	.779	.196	.001	
S7	Pearson correlation	-.027	.080^∗^	-.093^∗∗^	.006	.123^∗∗^	.061
	Sig. (2-tailed)	.425	.020	.006	.864	.000	.074
S8	Pearson correlation	-.016	-.101^∗∗^	-.068^∗^	-.055	-.014	-.023
	Sig. (2-tailed)	.633	.003	.049	.109	.692	.509
S9	Pearson correlation	-.087^∗^	-.111^∗∗^	-.078^∗^	-.015	-.018	-.034
	Sig. (2-tailed)	.011	.001	.024	.656	.610	.315
S10	Pearson correlation	.b	.b	.b	.b	.b	.b
	Sig. (2-tailed)	.	.	.	.	.	.

**Table 3:** Correlations ^d^ (b).

		S7	S8	S9	S10
S1	Pearson correlation	-.027	-.016	-.087^∗^	.b
	Sig. (2-tailed)	.425	.633	.011	.
S2	Pearson correlation	.080^∗^	-.101^∗∗^	-.111^∗∗^	.b
	Sig. (2-tailed)	.020	.003	.001	.
S3	Pearson correlation	-.093^∗∗^	-.068^∗^	-.078^∗^	.b
	Sig. (2-tailed)	.006	.049	.024	.
S4	Pearson correlation	.006	-.055	-.015	.b
	Sig. (2-tailed)	.864	.109	.656	.
S5	Pearson correlation	.123^∗∗^	-.014	-.018	.b
	Sig. (2-tailed)	.000	.692	.610	.
S6	Pearson correlation	.061	-.023	-.034	.b
	Sig. (2-tailed)	.074	.509	.315	.
S7	Pearson correlation	1	.006	-.021	.b
	Sig. (2-tailed)		.854	.537	.
S8	Pearson correlation	.006	1	.380^∗∗^	.b
	Sig. (2-tailed)	.854		.000	.
S9	Pearson correlation	-.021	.380^∗∗^	1	.b
	Sig. (2-tailed)	.537	.000		.
S10	Pearson correlation	.b	.b	.b	.b
	Sig. (2-tailed)	.	.	.	

^∗^Correlation is significant at the 0.05 level (2-tailed). ^∗∗^Correlation is significant at the 0.01 level (2-tailed). ^b^It cannot be computed because at least one of the variables is constant. ^d^List wise *N* = 851.

**Table 4:** Case processing summary.

		*N*	%
Cases	Valid	170	99.5
	Excluded^a^	4	.5
	Total	174	100.0

**Table 5:** Reliability statistics.

Cronbach's alpha	Cronbach's alpha based on standardized items	*N* of items
.962	.962	18

**Table 6:** Item statistics.

	Mean	Std. deviation	*N*
OnlineClassesHelpLongRun	-0.51	1.198	170
OnlineClassesWillImproveLearning	-0.55	1.162	170
PersonalSuccessByOnlineClasses	-0.44	1.181	170
OnlineClassesHelpBoostSkills	-0.61	1.132	170
OnlineClassesAreSimpleToUse	-0.39	1.212	170
OnlineClassesMoreFlexible	-0.62	1.166	170
FavorableAttitudeTowardsOnlineClasses	-0.48	1.198	170
OnlineClassesImpactsPositivityOnMe	-0.55	1.182	170
OnlineClassesUseIsTrend	-0.24	1.237	170
IntendToUseOnlineClasses	-0.43	1.191	170
IncreaseOccurracneOfOnlineClasses	-0.49	1.142	170
OnlineClassesWillEnhance	-0.54	1.255	170
OnlineClassesConsistentWithDevices	-0.35	1.204	170
SystemUseWillBoostMyLearning	-0.35	1.148	170
OnlineClassesMatchesWithOldSystem	-0.64	1.164	170
TryAnyFunction	-0.19	1.250	170
IknowBefore	-0.22	1.266	170
TryTechnologyToEvaluate	-0.08	1.285	170

**Table 7:** Interitem correlation matrix.

	OnlineClassesHelpLongRun	OnlineClassesWillImproveLearning	PersonalSuccessByOnlineClasses	OnlineClassesHelpBoostSkills	OnlineClassesAreSimpleToUse	OnlineClassesMoreFlexible	FavorableAttitudeTowardsOnlineClasses	OnlineClassesImpactsPositivityOnMe	OnlineClassesUseIsTrend	IntendToUseOnlineClasses	IncreaseOccurracneOfOnlineClasses	OnlineClassesWillEnhance	OnlineClassesConsistentWithDevices	SystemUseWillBoostMyLearning	OnlineClassesMatchesWithOldSystem	TryAnyFunction	IknowBefore	TryTechnologyToEvaluate
OnlineClassesHelpLongRun	1	0.789	0.757	0.683	0.577	0.633	0.590	0.614	0.526	0.656	0.588	0.712	0.626	0.605	0.547	0.470	0.454	0.415
OnlineClassesWillImproveLearning	0.789	1	0.744	.714	0.599	0.552	0.575	0.614	0.564	0.653	0.607	0.697	0.660	0.629	0.568	0.425	0.421	0.437
PersonalSuccessByOnlineClasses	0.757	0.744	1	.731	0.611	0.581	0.670	0.716	0.459	0.672	0.607	0.682	0.651	0.657	0.580	0.480	0.592	0.522
OnlineClassesHelpBoostSkills	0.683	0.714	0.731	1	0.568	0.579	0.653	0.629	0.510	0.656	0.605	0.626	0.605	0.607	0.612	0.491	0.555	0.462
OnlineClassesAreSimpleToUse	0.577	0.599	0.611	0.568	1	0.564	0.569	0.545	0.594	0.626	0.576	0.559	0.603	0.547	0.556	0.545	0.469	0.470
OnlineClassesMoreFlexible	0.633	0.552	0.581	0.579	0.564	1	0.697	0.665	0.546	0.624	0.618	0.640	0.576	0.550	0.588	0.439	0.42	0.329
FavorableAttitudeTowardsOnlineClasses	0.590	0.575	0.670	0.653	0.569	0.697	1	0.722	0.603	0.723	0.724	0.613	0.650	0.591	0.590	0.552	0.528	0.544
OnlineClassesImpactsPositivityOnMe	0.614	0.614	0.716	0.629	0.545	0.665	0.722	1	0.547	0.677	0.651	0.699	0.604	0.677	0.629	0.551	0.58	0.457
OnlineClassesUseIsTrend	0.526	0.564	0.459	0.51	0.594	0.546	0.603	0.547	1	0.622	0.555	0.517	0.544	0.483	0.437	0.511	0.413	0.565
IntendToUseOnlineClasses	0.656	0.653	0.672	0.656	0.626	0.624	0.723	0.677	0.622	1	0.785	0.700	0.715	0.654	0.662	0.522	0.460	0.534
IncreaseOccurracneOfOnlineClasses	0.588	0.607	0.607	0.605	0.576	0.618	0.724	0.651	0.555	0.785	1	0.646	0.662	0.576	0.617	0.499	0.528	0.477
OnlineClassesWillEnhance	0.712	0.697	0.682	0.626	0.559	0.640	0.613	0.699	0.517	0.700	0.646	1	0.665	0.591	0.590	0.528	0.447	0.464
OnlineClassesConsistentWithDevices	0.626	0.660	0.651	0.605	0.603	0.576	0.650	0.604	0.544	0.715	0.662	0.665	1	0.757	0.568	0.612	0.559	0.544
SystemUseWillBoostMyLearning	0.605	0.629	0.657	0.607	0.547	0.550	0.591	0.677	0.483	0.654	0.576	0.591	0.757	1	0.679	0.588	0.614	0.586
OnlineClassesMatchesWithOldSystem	0.547	0.568	0.580	0.612	0.556	0.588	0.590	0.629	0.437	0.662	0.617	0.590	0.568	0.679	1	0.502	0.410	0.447
TryAnyFunction	0.470	0.425	0.48	0.491	0.545	0.439	0.552	0.551	0.511	0.522	0.499	0.528	0.612	0.588	0.502	1	0.595	0.705
IknowBefore	0.454	0.421	0.592	0.555	0.469	0.420	0.528	0.580	0.413	0.460	0.528	0.447	0.559	0.614	0.410	0.595	1	0.596
TryTechnologyToEvaluate	0.415	0.437	0.522	0.462	0.470	0.329	0.544	0.457	0.565	0.534	0.477	0.464	0.544	0.586	0.447	0.705	0.596	1

**Table 8:** Scale item-total statistics.

	Mean if item deleted	Variance if item deleted	Corrected item Total correlation	Squared multiple correlations	Cronbach's alpha if item deleted
OnlineClassesHelpLongRun	-7.16	251.760	0.771	0.738	0.959
OnlineClassesWillImproveLearning	-7.12	252.661	0.771	0.756	0.959
PersonalSuccessByOnlineClasses	-7.23	250.817	0.809	0.780	0.959
OnlineClassesHelpBoostSkills	-7.06	253.298	0.775	0.672	0.959
OnlineClassesAreSimpleToUse	-7.28	253.257	0.720	0.572	0.960
OnlineClassesMoreFlexible	-7.05	254.341	0.720	0.646	0.960
FavorableAttitudeTowardsOnlineClasses	-7.19	250.714	0.800	0.730	0.959
OnlineClassesImpactsPositivityOnMe	-7.12	251.174	0.799	0.739	0.959
OnlineClassesUseIsTrend	-7.44	254.354	0.674	0.604	0.961
IntendToUseOnlineClasses	-7.24	249.924	0.827	0.768	0.958
IncreaseOccurracneOfOnlineClasses	-7.18	252.907	0.779	0.709	0.959
OnlineClassesWillEnhance	-7.14	249.893	0.782	0.692	0.959
OnlineClassesConsistentWithDevices	-7.32	250.514	0.801	0.731	0.959
SystemUseWillBoostMyLearning	-7.32	252.526	0.785	0.744	0.959
OnlineClassesMatchesWithOldSystem	-7.03	254.443	0.719	0.625	0.960
TryAnyFunction	-7.48	253.92	0.678	0.649	0.961
IknowBefore	-7.45	254.746	0.647	0.611	0.961
TryTechnologyToEvaluate	-7.59	254.551	0.641	0.671	0.961

**Table 9:** Scale Statistics.

Mean	Variance	Std. deviation	*N* of items
-7.67	282.494	16.808	18

## Data Availability

We are attaching dataset files that are used in this paper (dataset link: https://github.com/sobiawassan/The-Impact-of-Online-Learning-System-on-Students-Who-Affected-with-Stroke-Disease-main.git).

## Supplementary Materials

Supplementary Materials The impact of online learning system on students who affected with stroke disease.
